# Outcome Prediction of Hematologic Malignancy in Critically Sick People

This article has been retracted.

**DOI:** 10.1155/2022/3234484

**Published:** 2022-07-18

**Authors:** Palanivel Velmurugan, Vinayagam Moihanavel, Malik A. Altayar, Mohammed M. Jalal, Saeed M. Kabrah, Husam Qanash, Majed N. Almashjary, Osama M. Alshehri, Vijay Singh Kunwar

**Affiliations:** ^1^Centre for Materials Engineering and Regenerative Medicine, Bharath Institute of Higher Education and Research, Chennai, 600073 Tamil Nadu, India; ^2^Department of Mechanical Engineering, Chandigarh University, Mohali-140413, Punjab, India; ^3^Department of Medical Laboratory Technology, Faculty of Applied Medical Sciences, University of Tabuk, Tabuk, Saudi Arabia; ^4^Department of Laboratory Medicine, Faculty of Applied Medical Sciences, Umm Al-Qura University, Saudi Arabia; ^5^Department of Medical Laboratory Science, College of Applied Medical Sciences, University of Ha'il, Hail 55476, Saudi Arabia; ^6^Molecular Diagnostics and Personalized Therapeutics Unit, University of Ha'il, Hail 55476, Saudi Arabia; ^7^Department of Medical Laboratory Sciences, Faculty of Applied Medical Sciences, King Abdulaziz University, Jeddah, Saudi Arabia; ^8^Hematology Research Unit, King Fahd Medical Research Center, King Abdulaziz University, Jeddah, Saudi Arabia; ^9^Department of Clinical Laboratory Sciences, College of Applied Medical Science, Najran University, Najran, Saudi Arabia; ^10^Department of Biotechnology, Himalayan Whitehouse International College Address, Kathmandu 44600, Nepal

## Abstract

People with hematologic malignancies (HM) frequently postulate intensive care unit (ICU) hospitalization due to organ damage caused by the disease process or treatment-related consequences. This study is aimed at looking at mortality and sign factors in adult patients with hematologic malignancy (HM) who have been hospitalized in the ICU. Death was one quality indicator; researchers used a machine learning approach to find determinants of death. As per the study, there have been 206 patients hospitalized in the ICU (mean age: 51.3 ± 13.6 years; 60% male). The average length of stay was three days, with 14.1% requiring extended ICU commitment. ICU death was 45.6% at 30 days, 62.6% at sixty days, and 74.3% at twelve months, rising to 59.2% at thirty days, 62.6% at sixty days, and 74.3% at twelve months. Ventilation systems and vasodilating medication were linked to higher ICU death, but admission to the ICU surgically and experiencing malignancies are linked with lower death rates. Patients with HM who are hospitalized in the ICU have a high mortality rate (45.6%), which rises to 74.3% after a year. Serious illness, postsurgical hospitalization, and malignancy were revealed as determinants of patient outcomes in multivariate analyses.

## 1. Introduction

Hematologic malignancies are cancers that begin in blood-forming tissues, such as the bone marrow or immune system cells. Lymphoma, leukemia, and multiple myeloma are the three types of hematologic malignancies. Lymphoma is a cancer that starts in the lymphatic system, which is an integral part of innate and adaptive immunity. Leukemia is a blood cancer that begins in the bone marrow and spreads throughout the body. Multiple myeloma is cancer that attacks B lymphocytes and extends through the bone marrow. Invasion mold infections such as mucormycosis, aspergillosis, and fusariosis, which were less prevalent, are significant side effects of immunosuppressive drug treatment for malignant tumors [1]. People experiencing allogeneic hematogenic stem cell transfusion (HSCT) or remission-induction chemotherapy for acute myeloid myelodysplastic/leukemia sickness (AML/MDS) face a 20-fold increased chance of respiratory infection than those with preexisting lymphoma or myelodysplastic syndrome. Even though diagnostic breakthroughs and specific antimicrobial medications have enhanced the survivability risk in patients with invasive aspergillosis, about one-third of victims die from the disease or even have life-saving treatment interrupted while the mold disease is recognized. Consequently, several hematologists use blood galactomannan testing and high-resolution computed tomography aspects to evaluate patients for impending mold disease or prescribe mold-active antimicrobial prophylactic for extended periods if the individual has a temperature even though only a tiny percentage of individuals (4-12%) will get a mold infection [2].

The research of the etiology, evaluation, therapy, prognostic, and mitigation of blood illnesses is known as hematology. A med-tech performing the laboratory work that has gone through the examination of the blood is restricted, and most miniature cities and hospitals lack a specialist. As a result, this procedure can be pretty helpful, and it can be utilized in any medical center, facility, and even laboratory for essential evaluation before being submitted to hematologists. Initially, the researchers used a convolutional neural network to look for disorder classification and prognosis [3]. The research discovered that the most thorough research and approaches are rarely carried out throughout the medical field. Several convolutional neural networks were employed to diagnose certain illnesses. Tumor melanoma uses an elongated tissue sample; they developed and evaluated multivariate models forecasting prostate cancer with an initial biopsy and examined whether these long biopsy-based designs and a neural network that is contrasted with regression analysis to predict this melanoma, cardiovascular disease such as coronary heart disease. Intensive care began with the isolation of acutely unwell, preoperative individuals in a hospital waiting room where they had been closely monitored. As novel surveillance, therapy, and surgery methods became accessible, healthcare facilities enlarged their ICU, tightened admittance requirements, and relied more heavily on exceptionally trained personnel to provide healthcare. Research devised a severity of disease classification method to assess the preconception mortality risk in very ill patients to solve these issues with accuracy. Information from Acute Physiology and Severe Health Evaluation analysis indicates stable and robust connections between the severity of symptoms and subsequent likelihood of fatal injury from infectious illnesses frequently handled in surgical and medical ICU preceding multi-institutional and environmental studies. In individuals with cancer, neurological dysfunction is a common cause of death [4]. This would include malignant cell invasion of the central nervous or meninges, pathogens, cerebrovascular disease, and metabolic abnormalities that are not directly linked to cancer therapies or paraneoplastic disorders. Participation of the central and peripheral nervous system demanding charge of the ICU has been documented in up to 25% of people living with severely sick cancer. Nevertheless, no research has been carried out primarily to investigate the causes and consequences of neurologic disorders inside this community. Patients undergoing bone marrow transplants, particular malignancies, or specific patterns of problems were the subject of very few investigations of neurological occurrences in people living outside the ICU [5].

The specific neurodegenerative illness of the core sources requiring intensive care treatment for tracking or resuscitative maintenance was described as a neurologic breakdown. This included disturbance of consciousness, epilepsy both with and without epileptic seizures, focal signal encephalitis, and meningeal complaints. The lack of arousal and consciousness was classified as coma, measured using the Glasgow Coma Scale (GCS). Uncertainty, behavioral problems, changed level of awareness, and indications of emergency department or widespread neurologic noticeable symptoms were all used to characterize encephalopathy. Oncology individuals' admittance to the ICU has long raised concerns concerning both necessary and possible misuse of restricted resources. “Patients with hematological and biochemical or metastasizing to distant solid tumors are poor candidates for ICU admission, with a death frequency of up to 89.9%, according to the College of America of Critical Care Medicine Committee in 1999. It is recommended that initial therapy be limited or that ICU hospitalization be refused.” Nevertheless, data indicating relatively close ICU results (in the standing of death) for patients with solid tumors and, to a minor degree, hematoma oncological (HO) diagnosis has already been collected for a minimum of 15 years when compared with individuals lacking illness [6]. Survivors with malignant tumors have lived longer thanks to breakthroughs in detection, treatment, and palliative therapy during the last few generations. Victims who were enrolled in intensive care with malignant tumors, on the other hand, have a poor prognosis, with current statistics indicating up to 46 percent to 90 percent death rates in the in-hospital setting, which is significantly greater than the death rates of concurrent general medical confirmed cases enrolled to the ICU [7]. Various research has emphasized the requirement for antihypertensive drugs, ventilators, and the intensity of the disease as indicators of ICU death. Renal failure has been beneficial for severely ill cancer patients with noninvasive ventilators (NIV). In people living with hypoxemic cancer with respiratory failure, NIV improves oxygen for bronchoalveolar lavage and bronchoscopy and reduces the necessity for insertion. NIV also has been enhanced over the previous decade among people with cancer with respiratory failure and those who needed ventilatory assistance, decreasing insertion in almost half of the instances.

As a result, NIV is increasingly deployed in hypoxemic immunocompromised patients with high risk. Concerns were expressed about the adverse prognosis linked to long-term utilization of NIV and its potential ineffectiveness. Hematologic malignancies have become a significant concern to persons of different ages and have had a global impact on people's standard of living. Although the most up-to-date and effective chemotherapeutic medications for specific tumors are critical for improving the health outcomes of patients with hematologic malignancies, precise early identification should take precedence [8]. Biopsy, peripheral blood work, bone marrow biopsy, flow cytometry, chromosomal analysis, radiologic examination, immunology testing, and DNA sequencing technologies are modern tools and technologies used to diagnose hematologic malignancies. Due to the shortcomings of the previously mentioned clinical detection approaches, such as heavy price, time demand, complications, and nuclear contamination, it is interesting to make a novel consumer and expense technique with higher accuracy to identify hematologic cancers. NIV have become one of the most incredible significant advancements in ventilators throughout the last twenty years. Since the mid-1990s, the use of NIV in treating acute respiratory failure (ARF) has expanded for all indications, encompassing individuals either without or with chronic obstructive pulmonary sickness, saying there is no indication for either [9]. Furthermore, prognosis indicators differ according to the research agency's features, client demographic, the kind of HM, and the training regimen in only certain circumstances. Even though a lot of research has examined long-term consequences in HM patients admitted to the ICU, more research from various centers is required to confirm the conclusions of previous papers. In particular, data are scarce from the Canadian health system to inform the care of severely sick HM sufferers.

Hematologic malignancies have become a significant concern to persons of different ages and have had a global impact on people's standard of living. Although the most up-to-date and effective chemotherapeutic medications for specific tumors are critical for improving the health outcomes of patients with hematologic malignancies, precise early identification should take precedence. Biopsy, peripheral blood work, bone marrow biopsy, flow cytometry, chromosomal analysis, radiologic examination, immunology testing, and DNA sequencing technologies are modern tools and technologies used to diagnose hematologic malignancies [10]. Due to the shortcomings of the previously mentioned clinical detection approaches, such as heavy price, time demand, complications, and nuclear contamination, it is interesting to make a novel consumer and expense technique with higher accuracy to identify hematologic cancers. The microenvironment of blood cells is made up of a complicated web of cellular connections and exposure to various secreted substances. This milieu is found in stromal cells, osteoblasts, hematopoietic stem cells, osteoclasts, B and macrophages, T lymphocytes, and other inflammatory responses. There are two kinds of resistance in the immune response: adaptive and innate immune. The body's initial line of defense against pathogens is widely assumed to be an inherent autoimmune condition; nevertheless, the reaction to viruses is nonspecific. Adaptive immunity allows for a solid inflammatory system by recognizing “non-self” antigens and retaining the immunological response to infections encountered previously [11].

### 1.1. Related Work

The research is done to predict the rate and risk of hematologist malignancies. In this article, more than 1700 hospital data of nearly 800 patients' HM information were collected from 2005 to 2008. To process an unreasonable risk, multiple regression analysis is utilized. For a purpose, the total average jeopardy rating for internet movie database (IMDB) can precisely distinguish patients with HM who are at reduced risk for having a mild illness. It may be possible to “monitor out” low-risk sick people who are less positioned to gain from intensive diagnosing, tracking, or blemish antimicrobial activity prophylactic. This research provides the entire detail on the risk factor of HM and the design method with its ethics statement and data collection based on the study population and the study endpoint. The technique provides only the general concept of the risk factors. The regression algorithm analyzes the data in the experimental section and predicts the risk factor. Impacts of posaconazole prophylaxis were discussed in Results, and in Discussion, the benefits and limitations were generally specified. The research risk score was developed from retrospective information in a centralized site. Researchers were unable to adjust for “real-life” confounding variables like the use of antimicrobial prophylactic were considered the major limitation of the research. Furthermore, indeed the grade was established explicitly for hematopoietic stem cell transplantation (HSCT) participants. Medical risk variables for immunodeficiency such as transplant vs. host illness and corticosteroids, which are not included in the final evaluation method, might likely be much more significant. Indeed, the relative risk was to be used in the diagnosis and management of immunodeficiency at other clinics, comprehensive verification, and middle modification would almost certainly be needed for the research proposed by [12].

Cancer has been defined as a diverse disease through various subcategories. Past detection and prediction of a form of cancer have developed a requirement in cancer investigation. Subsequently, it can assist with outpatient therapeutic practice. The need to classify cancer patients into low- and high-risk groups has encouraged several biomedical and bioinformatics research organizations to look into using machine learning (ML) technology. As a result, these methods simulated the development and therapy of malignant conditions—the treatment of malignant diseases. Additionally, the ability of machine learning tools to find key features in complicated datasets demonstrates their value. Decision trees, Bayesian networks, artificial neural networks, and support vector machines are among the approaches extensively used in cancer charities to construct forecasting designs, resulting in reliable and time-made decisions. Even though it is evident that the utilization of machine learning techniques can assist the researcher in better understanding cancer growth, adequate testing should be done before these innovations can be applied to medical treatment. Research gives an overview of contemporary machine learning algorithms used in cancer development modeling in this paper. The forecast design is based on a supervised machine learning approach and various input variables and datasets. Given the increasing trend of using machine learning approaches in cancer research, researchers have compiled a list of the most current papers that use these approaches to assess cancer risk or health experience. The primary restraint of the study is the minor amount of datasets which is one of the most main constraints mentioned in the research reviewed in this study. When utilizing categorization schemes to simulate a condition, one of the essential requirements is that the train databases have substantial enough. An extensive database enables adequate division into training and test sets, resulting in acceptable estimate verification. When contrasted with developing a deep understanding, a limited training population can lead to miscommunications, while estimation methods yield unsteady and biased systems. It is self-evident that a larger sample of patients utilized to forecast mortality can improve the prediction model's generalization. The research is based on the application of machine learning based on cancer prediction and prognosis proposed by [13].

There is little information on ICU admittance determinants in immunocompromised patients. This research is aimed at finding the determinants of admission to a hospital in immunocompromised patients admitted to a hospital. From March 2009 and December 2015, our hospital retrospectively reviewed cohort research on 820 sequential hospitalizations of patients with malignant hematological diagnoses. For MLR analyses, a backward elimination selection procedure was used. We looked for evidence of an informed directive conversation or direction not to do cardiac resuscitation during stay (CPR). Specific illnesses were documented, and the total score was adjusted. The residential care study ethics office approved the institutional review, which was carried out in compliance with the Tri-Council rules for following an ethical practice. The Sunnybrook Experimental Investigative Committee waived written consent because this was a retrospective study. The major limitation of the study is no evidence that body mass index (BMI), toxicity as a reason for admission, illness histology, chemotherapy intent, cytopenia, recent chemotherapy, presence of leukemia, line of chemotherapy, albumin, or comorbidity index scores were linked to an increase in mortality, as reported previously. This could be due to the minor example extent of ICU hospitalized individuals in this study or the selective reporting associated with administering induction chemotherapy to people with symptomatic leukemia [11]. To prevent ventilatory support, critically unwell hematologic patients admitted with acute respiratory distress are now being treated with noninvasive breathing. On the other hand, a lack of noninvasive breathing may increase death. Future research was conducted to regulate the occurrence of noninvasive ventilation failure and the factors that influence it. Multivariate investigation suggests that breathing rate under noninvasive ventilation (NIV), longer time among admittance, the first use of noninvasive air flow, need for vasopressors or kidney transplant therapeutic, and acute respiratory distress pathophysiology were all inversely correlated with noninvasive ventilation malfunction. Noninvasive respiratory loss happens in half of the chronically unwell hematologic patients and is linked to a higher death rate. NIV dropout predictors could be utilized to help guide insertion procedures. The major limitation or disadvantage of the paper is they cannot say for sure that the delay was unnecessary or that starting sooner would have lowered the risk of failure. It is probable that the delayed start time now represents the hospital's slow degeneration, which may be due to the substantial morbidity and mortality with late-onset organ damage [10].

Clients with hematologic malignancies (HM) often include ICU hospitalization due to organ dysfunction caused by the progression of the disease or treatment-related consequences. This study is aimed at looking at death and clinical characteristics in elderly cases with HM who have been hospitalized in the ICU. During 2004 and 2014, a systematic documentation study among all elderly patients with HM was hospitalized in the ICU of Canadian tertiary hospital care. Death was one of the primary outcomes. To find determinants of death, researchers used logistic regression. Throughout the trial, 206 patients with HM were hospitalized in the ICU. The average length of stay was three days, but 14.1 percent project context ICU hospitalization. ICU mortality was 45.6 percent at one month, 62.6 percent at sixty days, and 74.3 percent at one year, rising to 59.2 percent at one month, 62.6 percent at sixty days, and 74.3 percent at one year. Ventilation systems and vasodilator medication were linked to higher intensive unit death, but enrollment in the ICU retrospectively and experiencing myeloma were strongly correlated with death rates. Persons having HM who are hospitalized in the ICU get significant morbidity and mortality (45.6%), which rises to 74.3 percent within a year. Severe sickness, postoperative hospitalization, and malignancies were revealed as indicators of clinical satisfaction in a multivariable analysis. The restrictions of a surveying analysis conducted at a solo center are apparent in this investigation. Our review covered a diverse population of patients, which may restrict the relevance of our findings. Because this data was not frequently documented throughout the trial, we have been unable to incorporate well-defined ICU assessment methods such as the Acute Physiology and Chronic Health Evaluation (APACHE) II or Sequential Organ Failure Assessment (SOFA) in your assessment [9].

## 2. Methodology

The research is about predicting the outcome of hematologic malignancies in critical conditions. Different datasets were collected from other hospitals to expect work related to chronic diseases for hematologic malignancies. Research could provide a clear idea of the prediction of HM based on the collected data. The basic concept of the research is to provide better accuracy and precision. Thus, the research comes under the field of acute diseases. Noninvasive hematologic malignancy is also included in this research. The patients with critical sickness with acute renal failure are shown in the NIV mechanical ventilation. Researchers wanted to know what factors contributed to NIV failure in chronically sick hematological individuals with respiratory failure. This research is aimed at looking at characteristics that forecast the outcomes in severely ill people with HM that needed to be enrolled in the ICU. The following section could first describe the noninvasive mechanism based on the data collected from the hospital and continue to the noninvasive area; the main topic of the research based on hematological malignancy is discussed based on the collected data.

### 2.1. Noninvasive

The patient data who received NIV for HM were gathered from the medical ICU of Saint Louis, Paris. The University Hospital of Saint-Louis has 650 beds, including 330 for people with cancer (nine departments). Approximately 100 hematological cases, 50 solid tumor patients, and more than 400 noncancer people are enrolled in the ICU each year. The age group was under 18 years old, and they had to be infected with the acquired immunodeficiency syndrome [10]. Allogeneic hematopoietic cell transfusion was also ruled out due to a recent study published by our lab that found no advantage from NIV within those individuals. People with an end-of-life choice status that precludes insertion and those who underwent NIV as a preoxygenation strategy before endotracheal were excluded from the study.  Table 1 shows ICU admission based on patient's characteristics.

In Table 1, the victim case characteristics based on the intensive care admission are mentioned. This table includes the patient's gender, age, duration of access, underlying malignancy based on its type, diagnosis stage, remission of malignancy, and enrollment in ICU, and the mean can be computed. In the table, NIV (F) denotes the noninvasive failure, and NIV (S) indicates the noninvasive success [12].

### 2.2. Data Collection

The information in Tables 1–3 was gathered retroactively from case victim records for every case. Overall, white blood cells were used to characterize leukopenia. Senior official anesthesiologists examined thorax radiography. The Logical System Degradation rating was produced to quantify organ dysfunction at admittance and during the first three intensive days. The Modified Critical Physiological Assessment II has evaluated disease severity at ICU enrollment [14]. Malignancies transferred to the ICU at the initial cancer stage, particularly at the moment of diagnosis or during the initial course of treatment, were considered inauguration malignancy. The ICU was identified using the criteria mentioned in Table 2—NIV session characteristics.

Furosemide 15 to 60 mg was given when physicians feared cardiac and respiratory failure. All victims' vital statistics were accessible at discharge from the hospital. In addition to the ventilation mentioned above, modes utilized, the breathing rate and peak flow during NIV, the duration from ICU enrollment and NIV initial use, and the length (hours and weeks) of NIV usage were documented. The PaO_2_/FIO_2_ proportion and the first to be reported. The prognosis of respiratory failure was confirmed, and the results of bronchoalveolar lavage and fiberoptic bronchoscopy detailed before. The term ARDS is established, as said before [15].

### 2.3. Hematologic Malignancy

This research was conducted at the Victoria General Hospital (VGH) of the Nova Scotia State Health Department in Halifax, Nova Scotia, Canada. The ICU is an 11-bed surgery unit those board-certified anesthesiologists manage. It is the central ICU in Nova Scotia for immunocompromised patients. The Nova Scotia Health Authority Research Ethics Board approved this study. A nonrandomized prospective evaluation of clinical documentation was carried out. From January 1, 2004, to December 31, 2014, we analyzed the medical records of all people (above 18 years) victims enrolled in the VGH intensive care with a confirmed diagnosis of HM.

### 2.4. Contributors

All people with chronic leukemia, multiple myeloma, lymphoma, and acute leukemia who had a recognized diagnosis were examined for enrollment. Patients, including an HM who did not meet any of these signs and symptoms, were analyzed in this section and were assigned to the “other” group. A manual assessment of a specialized document ICU admittance log was used to identify participants in the study. Chart evaluations were carried out by going over each research patient's medical records and extracting data into a single database created by the investigators [16]. To maintain the reliability of the findings, information from a victim's initial ICU admission has been included in the study if they had over than ones in that same hospitalization. The research team agreed that a two-year gap between ICU stays would be enough time to distinguish between observation and analysis for almost the same victim. As a result, data for case victims who were enrolled in the ICU several times over more than two years were deemed multiple data groups.

### 2.5. Data Collection

Health records, ICU admittance, diagnosis, duration of ICU hospitalization, ICU relapse, kind of bone marrow aspiration, kind of HM, nonocclusive illness or febrile neutropenia, the prevalence of graft vs. host syndrome, sepsis or steroid utilization, and indication for steroid use were all obtained. Analytical factors included the majority of neutropenia, anemia, or thrombocytopenia on admittance to the ICU and the prevalence of disease before to or during hospitalization [9]. Blood and infection were considered unless positive cultures were confirmed in wound swabs, catheter tips, urine, sputum, or bronchial washings. During the ICU hospitalization, the need for function maintenance was demonstrated by utilizing vasopressors and mechanical breathing, inotropes, and hemodialysis. Just information from the health record was gathered. Data that was not accessible was marked as unavailable, and no information was substituted in its place.

### 2.6. Characterizations

The scientists classified the diagnosis based on what they considered the most severe problem is needing ICU hospitalization. Neurological, renal, hemodynamic, postoperative, respiratory, and follow-up post-cardiopulmonary failure was utilized to identify admission diagnoses in the intensive care unit. The term “breathing” was described as the need for ventilatory support, including noninvasive and invasive mechanical ventilation [17]. Individuals who had a lower state of consciousness reported in the medical record on admittance to the ICU were classified as “neurological” (e.g., cerebrovascular and seizure incidents). ICU admittance for the necessity of kidney replacement therapy during ICU admission was classified as “renal.” “Hemodynamic” is necessary for ICU admission due to hypoglycemia requiring vasopressor and inotropic support or invasive tracking that could never be performed in the clinic. Victims undergoing ICU hospitalization following an approved protocol caused by a consequence of their HM were classified as “postoperative.” Victims transferred to the ICU after an incident on the ward were considered “follow-up post-cardiopulmonary arrest” [18].

### 2.7. Analysis of Data

Age, gender, category of HM, prognosis, intensive care unit, duration of service, intensive care unit, previous transplantation of stem cells, readmission, steroid use before ICU hospitalization, and the existence of anemia on ICU admission, febrile neutropenia, thrombocytopenia, neutropenia, graft versus host disease, or infection were all evaluated utilizing descriptive and inferential statistics (percentages, means, standard deviation, and variance). The relationship between victim variables and outcomes was investigated using a logistic regression model (mortality). People with lymphoma, chronic leukemia, myeloma, and acute leukemia were compared with patients with every other kind of HM as a control group [19]. Wald's analysis was used to measure the impact of the logistic regression model. All analyses were different and statistically varied. A significant difference was defined as a probability value of less than 0.05. We use a probability value of more than 0.05 as an acceptable fit for the Hosmer-Le Cessie test to evaluate the designs' goodness of fit [19].

At the beginning of the survey, the majority had been in their 6th or 7th generation, 19 were male, and the majority lived with such a relative, with three residing independently. There were ten cases of CLL myeloma, eight issues of FL, and five instances of MZL in the group of 12. Rich data was gathered, and a reflective conceptual finding shows four significant themes and eleven subtopics [13]. The following were some of the major themes: (1) incurable yet treated, (2) knowledge and awareness of chronic blood cancers, (3) treatable (but still incurable), and (4) future uncertainty, impact on sufferers. Each theme is broken down into subthemes. Italicized quotes are linked to participant numbers (e.g., P_1_ for the client and P1R for the patient's relatives) and diagnosis. The hierarchy of themes and subthemes is depicted in Figure 1.

#### 2.7.1. Theme 1

*(1) Distress Relief*. This topic depends on the data supplied by health professionals to increase patient and family comprehension of the features of persistent hematologic malignancies and a comment a thread on how to respond to them. Patients commonly expressed dissatisfaction with HCPs who described their malignancy as terminal but curable [20].

#### 2.7.2. Theme 2

*(1) Progression*. Patients were warned that while advancement was unlikely, it might occur at any moment and on countless occasions, necessitating several rounds of progressively intense treatment. Modifications were claimed to occur gradually or quickly, and they can somehow result in treatment regimens being changed. P_18_ (myeloma), for instance, recalled steadily “growing increasingly exhausted” as he recovered inside the posttransplant time, with additional chemotherapy administered before the scheduled second transplantation, which had been abrupt as his “free light chain had soared right back immediately” [13].

*(2) Prognosis*. Victims said they were informed that their life expectancy was likewise uncertain when it came to a diagnosis. Interestingly, there was acknowledgment and acceptance that something like this represented genuine clinical uncertainty instead of hiding information caused by unexpected malignancy [21]. This patient seems to grasp that specialists cannot be confident about particular patients, and nobody can know what is ahead.

#### 2.7.3. Theme 3

As indicated in the subthemes underneath, possessing a curable but irreversible persistent hematologic malignancy impacted differential evolution. The prognosis increased or lost significance over time, and some patients endured significant emotional challenges managing unknown outcome routes.

*(1) Diminishing Impact*. Several people became acclimated to having apathetic leukemia as they got accustomed to it, particularly if they would not have needed therapy but were being checked less frequently. This became especially evident in chronic lymphocytic leukemia (CLL) and to a smaller extent in other diseases, including one patient (P_26_, myeloma) commencing with 90 days of screening and then reducing to six monthly checks before getting substituted by a conference consultation [22].

*(2) Emotional Difficulties and Impact*. A persistent hematological malignancy has a profound impact on many people's lives. Patients in one group looked to be experiencing extreme mental discomfort, which was giving them more trouble than cancer's physical ailments.

*(3) Survival*. Chronic blood malignancies, despite becoming curable, were usually regarded as incurable, which can affect mortality, which was a source of anxiety for some, especially the young individuals such P_28_ [23].

#### 2.7.4. Theme 4

*(1) Unexpected Treatment*. Some patients had been diagnosed by chance and thought they were in good health, but they were taken aback when they learned they had a malignancy. P_21_ was identified “by chance” during a routine inspection of individuals with myeloma, while P_16_ stated his symptoms started “out of the blue” because he thought himself healthy and energetic [24]. Others would have only mild symptoms and did not invariably feel sick, such as P_22_ (CLL), who was surprised to be informed that he was “a very shoddily man” at his initial consultation because his only previous sign was tired all the time; P_15_ (FL), who declared “I was just not sick was the mounds I found”; and P_27_ (CLL), who said he felt much better except for mobility problems. Some individuals have exacerbated this since they had gone to the doctor because of what researchers thought were unconnected ailments, eventually linked to their blood malignancy [25].

*(2) Former Data*. Several patients indicated they seemed to have no idea what form of cancer they have, including one who admitted that he thinks of “normal cancer” but just not myeloma (P_16_). P_13_ stated that she knew “anything” regarding CLL, whereas P_29_ claimed that she knew leukemia was a “blood cancer,” but that was it. P_30_ admitted that he “had not ever heard of myeloma before I visited the doctor” [25]. Victims who did sometimes not consider the characteristics of their persistent blood cancer originally reported concentrating on specific words like “not curable” and “leukemia,” which may be distressing, causing panic and fear, mainly because there was little consciousness regarding dissolute and symptomatic subgroups or the various paths and consequences that come with every one of these.

*(3) Chronic Blood Cancer Expectation*. Many people were perplexed by their cancer's features and how it could not just be eliminated. P_5_ (MZL) defined her most significant hurdle in this regard as the fact that what appeared to be a gastrointestinal condition cannot be addressed with such a simple “zap”; the researcher could, however, recognize that her tumor was not the kind that might simply be “getaway of.” Correspondingly, P_13_ (CLL) said it was difficult for the researchers to recognize that they had leukemia. However, the first sign was a lump in the armpit, which also did lead them to believe that “if it were a lump, they could just consider taking it out,” which would have been a “bit of shock” when she discovered it was not feasible because the melanoma was in the blood [26].

Most patients were due to commence treatment immediately after they were diagnosed, understanding the relevance of prior malignancies, while most were initially examined. Although this may have delighted many, especially if an HCP had plainly stated reasoning, many people have found it harder to understand. “It is hard to grasp, you possess something disturbing when nothing occurs,” remarked P_26_ (myeloma). P_15_ (FL) says they found it challenging to comprehend and accept this fact because they were “unprepared” for this. They were also unsure about the instances that would direct her beginning diagnosis and said, “that has always been a concern.” They said that how a physician would recognize when and where to take the medication: it was almost as if you must become sick [27].

*(4) Lack of Knowledge*. Although some people eventually understood their sickness, some did not appear to get there and remained unsure about their cancer decades back. P_32_, in contrast, stated that she was unable to share her prognosis with their families because they did not fully comprehend: “They have still never.” “They have a son and a daughter, but they have not informed” them since they do not understand their situation. P_20_ said he notified his family members but not his acquaintances because he did not think they would comprehend how the treatments had not begun: “I do not advertise it.” P_25_ reiterated this sentiment, claiming that people are unaware of the features and consequences of malignancy [28].

*(5) Relapse and Progression Sign*. Numerous clients displayed a thorough understanding of the indicators of progress monitoring, as well as how to react to them. “When I feel any B signs of sleep disturbances, skin exhaustion, you have respiratory difficulties and everything, I keep a close eye out and call them (HCPs).” (P_34_: FL) and P_25_ (FL) stated that they would “know right away whether something was incorrect.” Some, on the other hand, were concerned about their low level of awareness. For instance, P_19_ (FL) stated that she was not instructed what to look for at first and was “not confident that I always know if was back.” It was challenging for some to be in charge of identifying potential indicators of advancement and selecting whether to disclose them, such as P_35_ (myeloma) [29].

## 3. Results and Discussion

Based on the research process, 509 hematological individuals suffering from ARF were transferred to the intensive care unit, with 113 meeting the report's eligibility requirements. The actual cohort consists of 99 patients, while information on NIV was lacking in 14 of them. Case victims who failed NIV required greater vasopressors and hemodialysis during the period they were getting NIV, as seen in Table 3. Individuals who underwent intubation used to have a considerably higher day 2 and day 3 logistic system degradation score, even though their logistic organ dysfunction point tally was not statistically different at admission. In addition, only one of the patients diagnosed with the renal disease did not involve insertion or MV.

Table 3 shows the outcomes of the NIV-based MLR system design. Researchers used a multivariate logistic regression approach (forward technique) to find the predictive factors of NIV (F) by utilizing the MV (i.e., failure of NIV) as the findings of the outcome variable, as evaluated by calculating odds ratios (OR) with the confidence interval of 95 percent (CI). Factors that yielded *ρ* the value of 0.10 in the univariate examination were included in the multiple regressions.

Figure 2 shows a flow diagram illustrating the study contributor selection procedure. Between 2004 and 2014, 204 adult cases with hematologic malignancies were hospitalized in the intensive care unit. Among these, victims were hospitalized in the ICU during the sample period, and every one of these hospitalizations was treated as a unique case. There have been 206 instances of HM during the study that required ICU hospitalization.  Table 4 shows the features of these 206 instances.

### 3.1. ICU

Table 5 shows the treatments performed on HM patients in the ICU. In 148 instances, evacuation and endotracheal intubation were necessary (71.7 percent). In 117 cases (56.9%), vasodilator treatment was required, and dialysis was essential in 35 patients (17.5 percent).

Figure 3 shows the ICU course factor involvement based on the four factors; they are reintubation which is denoted as a blue bar with minor cases and then hemodialysis, which is represented as a brown bar with minimum issues; mechanical ventilation has nearly 70% of cases dues to renal failure which is denoted as the gray bar, and finally, the yellow bar represents the vasopressor therapy with 585 of cases.

### 3.2. Outcomes of Patients

Table 6 shows the results of HM cases enrolled in the ICU. The table's graphical representation is mentioned in Figure 4. Following ICU enrollment, 45.6 percent of people died (94/206), as contrasted to 11.9 percent of all victims enrolled in this ICU throughout the research study. 59.3 percent (122/206) of HM patients who survived their ICU stay died within one month, and 74.5 percent (153/206) died within a year.

Table 7 and Figure 5 show the mortality rate for patients with a variant form of HM. Patients with severe leukemia brought to the ICU had the most significant risk of ICU mortality, at 64.3 percent (9/14). Patients admitted with multiple myeloma had the lowest rate of ICU death (4/21; 19.1%). Victims who had previously received a stem cell transplant had a 43.5 percent (40/92) ICU death rate and a 66.3 percent (61/92) 12-month fatality rate.

Table 8 shows the results of a logistic regression model used to find indicators for HM cases enrolled in the intensive care unit. According to the logistic regression model, vasopressors and mechanical ventilation in the ICU were linked to higher ICU death was shown in Figure 5. The utilization of vasopressors was still related to 1-month and two-month mortality, but not to one-year death rates. The Hosmer-Le Cessie test was inconsequential for many logistic regression analyses, suggesting no considerable challenges to the forecasting model's suitability. Furthermore, most variance inflation factors were less than two, indicating that the variables' occurrence was not a problem.

## 4. Discussion

Another of the most extensive Canadian-based studies of results in hematologic malignancy confirmed cases in the ICU in this research. The findings of this 10-year retrospective assessment show a significant rate of death (45.5%) in HM patients who required ICU hospitalization, comparable to 11.8 percent of the overall population in the same ICU. Surprisingly, deaths among HM patients who experienced ICU hospitalization increased to 74.5 percent after one year. Although examining many characteristics to predict patient outcome in ICU hospitalization, only vasopressor and mechanical ventilation were linked to higher ICU death rates, even though preoperative hospitalization and multiple myeloma were associated with higher survivability. In many facilities, admittance to the ICU is a significant investment in inpatient care and a restricted asset. Patients with HM have indeed been proven to demand higher expensive medication treatments in the ICU in aggregate. Nevertheless, the Ethics Committee of the French Society of Hematology recently established recommendations on the admittance of patients with hematologic malignancy to the intensive care unit, recommending whenever an HM patient arrives with organ damage, an interdisciplinary strategy involving the hematologist and intensivist should be used.

## 5. Conclusion

The inherent limitations of prospective data analyzed at a centralized location were overcome in this research. This report summarizes a diverse variety of patients, which might also restrict the relevance of our findings. Because this data was not frequently documented throughout the trial, we have been unable to incorporate well-defined ICU rating systems such as the APACHE II or SOFA in this assessment. According to this research, NIV failure is linked to latency in starting NIV with greater certainty in the intensive care unit. Nevertheless, the researcher cannot say for sure that the delay was unnecessary or that starting sooner might have lowered the likelihood of default. The later start time probably represented the patient's slow deterioration, which may be due to the deaths associated with delayed organ dysfunction. The paper could provide complete details on the hematological malignancy and outcome prediction based on the people admitted to the ICU and other wards. Even though various relevant variables were examined, only severe sickness, postoperative pain, hospitalization, and multiple myeloma were significant predictors of clinical outcomes. Based on the results of our analysis, researchers found that past dialogue among patients and caregivers about potential repercussions if they seek ICU hospitalization is critical. As they assist in administering the patient population, more study is needed to establish prognostic indicators. In conclusion, the regression analysis was used to make a prediction about the outcomes for the patients who had been diagnosed with hematological cancer. The prognosis for hospitalized severely sick individuals diagnosed with HM is getting better overall. However, the prognosis remains dismal for patients who are dependent on artificial breathing or who have undergone allogeneic heart-lung transplantation.

## Figures and Tables

**Figure 1:** Theme and subtheme hierarchical map.

**Figure 2:** Contributor selection.

**Figure 3:** ICU course factor.

**Figure 4:** ICU patient outcome.

**Figure 5:** Long-term and ICU death rate.

**Table 1:** ICU enrollment based on patient characteristics.

Case detail	NIV (F)	NIV (S)	*ρ*
Gender	40	30	0.25
Age	58	60	0.75
Use of tobacco	21	18	0.98
Past cardiac insufficiency	3	5	0.42
Causal malignancy			0.94
Leukemia	23	19	—
Non-Hodgkin lymphoma	15	14	—
Multiple myeloma	8	7	—
Severe myelogenous leukemia	1	1	—
Severe lymphocytic leukemia	8	5	—
Malignancy diagnosis	212	224	0.78
Malignancy remission	5	4	0.22
Hospital to ICU enrollment	10	9	0.46
Duration of symptoms	4	6	0.80

**Table 2:** NIV session characteristics.

Case detail	NIV (F)	NIV (S)	*ρ*
The duration between the enrollment in ICU and NIV	0	0	0.02
NIV duration in days	3	3	0.06
NIV duration in hours	9	9	0.49
Intake pressure support	13	13	0.28
Exhale pressure support	6	4	0.36
NIV respiratory rate	33	27	0.03
Tidal volume/weight	9.5	10.8	0.68

**Table 3:** MLR outcome with NIV (F).

	Odds ratio	Confidence interval	*ρ*
NIV breathing rate	1.19/point	1.06-1.34	0.006
Adjournment from ICU enrollment to NIV	3.00/day	1.03-3.95	0.05
Vasopressor requirement	6.52	1.60-26.54	0.008
Renal replacement therapy requirement	18.32	1.98-168.66	0.02
Criteria	77.72	6.89-878.39	0.0005

**Table 4:** Contributor study.

Representative	*n* = 206 cases
Age	51.2 ± 13.4
Gender	59.8%
Type of hematologic malignancy	—
Acute leukemia	34.6%
Lymphoma	33.6%
Chronic leukemia	6.9%
Myeloma	10.3%
Other	15.2%
Admission diagnosis	—
Hemodynamic	38.4%
Postarrest care	3.5%
Postoperative	8.4%
Neurologic	7.9%
Metabolic	2.5%
Respiratory	1.1%
Readmission	13.2%
Infection on admission	71.9%
Veno-occlusive disease	8.8%

**Table 5:** Involvement course in intensive care unit.

Factors	Cases
Reintubation	5.4%
Hemodialysis	17.5%
Mechanical ventilation	71.7%
Vasopressor therapy	56.9%

**Table 6:** ICU patient outcome.

Findings	Cases
ICU death rate	45.5%
One-month death rate	59.3%
Two-month death rate	62.5%
One year	74.5%

**Table 7:** Long-term and ICU death rate.

HM	ICU death	One-month death rate	Two-month death rate	One-year death rate
Chronic leukemia	64.4%	71.5%	78.5%	85.6%
Myeloma	19.2%	28.5%	28.5%	42.8%
Acute leukemia	49.4%	63.5%	69%	80.4%
Lymphoma	50.8%	63.9%	66.8%	75.4%
Other	35.6%	54.9%	54.9%	74.5%

**Table 8:** Prediction of logistic prediction of ICU and long-term death rate.

Predictor	Mortality of ICU	1-month of mortality	2-month of mortality	1-year of mortality
Age	1	1.03	1.03	1
Gender	0.84	0.93	1.2	1.53
*Malignancy*				
Chronic leukemia	3.34	1.9	2.8	1.47
Myeloma	0.5	0.26	0.23	0.19
Acute leukemia	1.23	1.36	1.88	1.38
Lymphoma	1.93	1.46	1.57	1.06
Other	1	1	1	1
Hemodynamic diagnosis	1	1	1	1
Mechanical ventilation	3.43	2	1.68	2.92
Hemodialysis	0.98	2.3	2.56	1.52
Vasopressor therapy	3.74	1.22	2.15	1.53

## Data Availability

The data used to support the findings of this study are available from the corresponding author upon request.
